# A Rare Presentation of Amlodipine-Induced B-Cell Pseudolymphoma: Case Report and Discussion

**DOI:** 10.7759/cureus.78140

**Published:** 2025-01-28

**Authors:** Juliana M O'Reilly, David S Kirwin, Travis Frantz, Vikas Shrivastava

**Affiliations:** 1 Medical School, Uniformed Services University of the Health Sciences, Bethesda, USA; 2 Department of Dermatology, Naval Medical Center San Diego, San Diego, USA

**Keywords:** amlodipine, b-cell cutaneous pseudolymphoma, cutaneous lymphoid hyperplasia, drug-induced, lymphoproliferative disorders

## Abstract

B-cell cutaneous lymphoid hyperplasia (CLH), or B-cell pseudolymphoma, is a benign lymphoid proliferative disorder that can mimic cutaneous lymphoma. This case describes a rare instance of amlodipine-induced B-cell pseudolymphoma in a 64-year-old woman. The patient presented with itchy papules and nodules on her neck and arms, occurring shortly after starting amlodipine for hypertension. Clinical examination and punch biopsies revealed lymphoid follicles with B-cell predominance. Gene rearrangement studies were negative for clonality, supporting a benign process. The patient’s reassuring clinical presentation, medication history, immunohistochemical staining and gene rearrangement analysis led to a diagnosis of B-cell CLH. Following the discontinuation of amlodipine lesions showed slow regression. Prior reports have described amlodipine-associated T-cell lymphoma but the literature lacks reports of amlodipine-induced B-cell pseudolymphoma. The diagnostic challenge lies in distinguishing pseudolymphoma from true lymphoma, emphasizing the importance of history, histopathological evaluation and clinical correlation.

## Introduction

This case study focuses on a 64-year-old woman presenting with pruritic papules and nodules, leading to a diagnosis of B-cell cutaneous lymphoid hyperplasia (CLH), also known as B-cell pseudolymphoma. Cutaneous pseudolymphomas are a group of rare conditions that can be triggered by various factors, including medications, and can closely resemble true lymphomas, necessitating careful diagnostic evaluation [1]. They are classified based on lymphocyte predominance though there are approaches that use histologic and clinical presentation for classification [1,2]. Diagnosis involves exploration of the patient's clinical presentation, medical history including infectious exposures (Borrelia burgdorferi species, HIV and syphilis), injections, arthropod bites, tattoos, and medications (anticonvulsants, antipsychotics, antihypertensives, antiarrhythmics, antibiotics, antirheumatics, anxiolytics, nonsteroidal anti-inflammatory drugs (NSAIDs)) [2]. Diagnostic work-up includes obtaining tissue biopsy for histopathologic analysis, immunohistochemistry staining, and gene rearrangement analysis. Depending on clinical suspicion further screening for infectious etiologies may be indicated [2]. The challenge of diagnosing pseudolymphoma stems from its similarities to other inflammatory conditions and lymphomas, the most concerning being lymphomas [1,2]. This report will explore the clinical presentation, diagnostic workup, and management of drug-induced B-cell pseudolymphoma. Based on an extensive review of the PubMed database, we are not aware of any other reported cases of amlodipine-induced B-cell lymphoma. We present this case in light of the limited available literature on the subject.

## Case presentation

A 64-year-old woman with hypertension, asthma, gastroesophageal reflux disease, and a distant history of cerebrovascular accident visited the dermatology clinic for a one-year history of itchy bumps on her neck and arms. Her medications included amlodipine (which she started three to four weeks prior to onset of cutaneous symptoms), levetiracetam (started approximately two to 2.5 years prior to onset of cutaneous symptoms), aspirin, atorvastatin, baclofen, cetirizine, omeprazole, and metoprolol. Review of systems, family, and social history were non-contributory. She denied vaccinations, tattoos, piercings, infections or insect bites in the weeks to months preceding her eruption. Examination revealed nine 2-millimeter to 1-centimeter multifocal smooth flesh-toned to red papules and nodules on her trunk and upper extremities (Figures 1, 2). The cervical, supraclavicular, axillary, inguinal, and popliteal lymph node examinations were normal.

**Figure 1:** Physical exam findings - Anterior neck and chest (A), Right forearm (B), Left upper extremity (C) Scattered nodules and papules on the anterior neck and chest, the largest being the 1 cm well-circumscribed firm red nodule with surrounding erythema on the left anterior neck (A). 5 mm well-circumscribed firm pink papule on the right dorsal forearm (B). Multiple scattered red papules on the dorsal left arm (C).

**Figure 2:** Dermoscopy findings: Left anterior neck (A), Right forearm (B) Dermoscopy findings of the left anterior neck nodule revealed a well-circumscribed red nodule with areas of brown pigmentation and surrounding erythema and pigmentation (A). Right dorsal forearm papule revealed a well circumscribed pink papule with central hypopigmentation, rim of brown pigmentation and areas of overlying white scale (B).

Punch biopsies revealed lymphoid follicles with tingible body macrophages in the dermis with B-cells reactive for CD20 and PAX5, germinal centers positive for CD10 and Bcl-6, negative for Bcl-2, and mild focal reactivity to CD30 (Figures 3, 4). CD21 (not pictured) demonstrated an intact follicular dendritic cell meshwork. Gene rearrangement analysis by polymerase chain reaction was negative for immunoglobulin clonality. Screening chest X-ray, HIV, syphilis and Lyme disease serologies were negative. The patient’s reassuring clinical presentation, medication history, immunohistochemical staining and reassuring gene rearrangement analysis led to a diagnosis of B-cell CLH, otherwise known as B-cell pseudolymphoma. 

**Figure 3:** Histology findings - Left anterior neck lesion H&E demonstrated superficial and deep dermal lymphoid infiltrates recapitulating lymphoid follicles. On higher power view of a representative follicle we can appreciate a normal follicular architecture and presence of tingible body macrophages. Ki-67 staining highlighted proliferative germinal centers in these follicles.

**Figure 4:** Histology findings - Left anterior neck lesion Immunohistochemical staining characterized lymphocytes within germinal centers as CD10, CD20, and Bcl-6 positive with negative staining for Bcl-2.

Our patient received intralesional steroids to her larger nodules. In addition, we noted slow regression of untreated lesions the following few weeks after discontinuing amlodipine, supporting the diagnosis of amlodipine-induced B-cell pseudolymphoma.

## Discussion

Pseudolymphoma is a benign lymphoid proliferative process that can mimic B- or T-cell lymphoma, triggered by stimuli like drugs, insect bites, infections, or foreign agents, though many cases are idiopathic [1,2]. 

Historically, there have been various classification systems used to describe these processes, with a recent report by Mitteldorf et al. proposing the separation of subtypes. They suggested four classifications: nodular, simulators of mycosis fungoides, other pseudolymphomas, and intravascular pseudolymphomas [1,2].

B-cell pseudolymphoma typically presents as solitary, red to purple nodule(s) under 4 cm on the face and upper thorax, more commonly in men under 40 [1-3]. Early biopsy and lymphocyte clonality analysis are helpful in distinguishing cutaneous lymphomas such as primary cutaneous follicle center lymphoma and primary cutaneous marginal zone lymphoma [1,2]. Histologically, there are nodular or diffuse intradermal collections of dense B-lymphocytes without significant nuclear atypia, along with reactive germinal centers, tingible body macrophages, and scattered plasma cells [1,2]. Occasionally there may be eosinophils or neutrophils present, and less than 30% have admixed T cells [1,2]. They display a polytypic pattern in immunoglobulin (Ig) light chain staining, a polyclonal Ig heavy chain, and have a high proliferation rate confined to the germinal center [1].

When encountering cutaneous B-cell infiltrates with a follicular growth pattern there are several factors which, when present, favor a benign process. They include the presence of tingible body macrophages within follicles (indicating normal apoptosis was occurring), increased proliferation within germinal centers, follicular cells staining negative for Bcl-2, and polyclonality on gene rearrangement analysis [4]. For use as a diagnostic distinguisher, both B-cell pseudolymphomas and B-cell lymphomas have variable clonality, so these findings should be considered within the entire clinical and histological picture [2,5].

Given clonality studies cannot completely distinguish pseudolymphoma from true lymphoma, there is risk of diagnosing a patient with pseudolymphoma when in fact they have burgeoning true lymphoma especially if original clonality studies were positive [5]. Furthermore, the same antigenic stimulation that caused cutaneous pseudolymphoma, if not removed, may continue to cause local inflammation and progress into true lymphoma [5]. This highlights the need for close follow-up with these patients. 

Drug-induced CLH has been reported in association with medications like phenytoin, amlodipine, fluoxetine, and carbamazepine with most cases showing T-cell predominant infiltrates or mixed T and B cells (81.5% and 10.5% respectively) [6].

The time interval between drug initiation to cutaneous findings is highly variable, ranging from 1-7300 days (shortest with antidepressants and longest with immunomodulators) with a median interval of 120 days [6]. The most common skin symptom was pruritus (59.2%), although 35.1% of patients were asymptomatic [6]. The median interval time from discontinuing the drug and recovery was 32.5 days [6]. Reported cases of amlodipine-induced T-cell pseudolymphoma resolved between three weeks and two months after discontinuation of the drug [7-9]. The most commonly reported medications associated with B-cell pseudolymphoma include valproate, atenolol, griseofulvin, imatinib, angiotensin-converting enzyme inhibitors, allopurinol, cyclosporine, levofloxacin, antihistamines, selective serotonin reuptake inhibitors (SSRIs), and phenytoin [3]. 

Though the exact pathogenesis of drug-induced pseudolymphoma is unknown, some authors postulate that implicated drugs may weaken immune function by interfering with immunosurveillance and subsequently abnormal lymphocyte proliferation [6,10]. For example, calcium channel blockers halt the potassium efflux in lymphocytes and beta-blockers impair the immunosuppressive role of norepinephrine on lymphocyte adrenoreceptors [6]. Although amlodipine is a well-known trigger for cutaneous pseudolymphoma, current studies solely describe amlodipine-induced T-cell pseudolymphoma [6-8]. To our knowledge, there are no reported cases of amlodipine-induced B-cell lymphoma (although there are cases of amlodipine-induced T-cell lymphoma). 

Treating the underlying cause, or removal of the offending agent for drug-induced cases followed by close monitoring for potential progression to true lymphoma are paramount [5,9,11]. Local treatment with cryotherapy, topical or intralesional steroids, laser, surgical excision or radiation have been employed [1]. For widespread lesions, systemic immunosuppressants may be considered [1,3].

This case has several limitations, including the potential for other contributing factors beyond amlodipine, a slower-than-expected regression of lesions and a short follow-up period for monitoring outcomes. These factors underscore the need for further studies to better understand the relationship between medications and cutaneous lymphoproliferative disorders.

## Conclusions

In conclusion, this case highlights the importance of a thorough understanding of the histopathological features and clinical context in differentiating between benign and malignant processes. Successful management of drug-induced cutaneous pseudolymphoma hinges on the timely identification and discontinuation of the offending agent, alongside appropriate treatment modalities for symptomatic relief, such as intralesional triamcinolone. In our case, follow-up was essential to continue evaluation of nodule regression and symptomatic management with intralesional triamcinolone. We also highlighted the importance of continued monitoring with our patient due to the known low risk of progression from cutaneous pseudolymphoma to true lymphoma. 

## References

[1] Mitteldorf C, Kempf W (2017). Cutaneous pseudolymphoma. Surg Pathol Clin.

[2] Mitteldorf C, Kempf W (2020). Cutaneous pseudolymphoma-a review on the spectrum and a proposal for a new classification. J Cutan Pathol.

[3] Khalil S, Donthi D, Gru AA (2022). Cutaneous reactive B-cell lymphoid proliferations. J Cutan Pathol.

[4] Leinweber B, Colli C, Chott A, Kerl H, Cerroni L (2004). Differential diagnosis of cutaneous infiltrates of B lymphocytes with follicular growth pattern. Am J Dermatopathol.

[5] Bergman R (2010). Pseudolymphoma and cutaneous lymphoma: facts and controversies. Clin Dermatol.

[6] Etesami I, Kalantari Y, Tavakolpour S, Mahmoudi H, Daneshpazhooh M (2023). Drug-induced cutaneous pseudolymphoma: a systematic review of the literature. Australas J Dermatol.

[7] Pulitzer MP, Nolan KA, Oshman RG, Phelps RG (2013). CD30+ lymphomatoid drug reactions. Am J Dermatopathol.

[8] Cheong KW, Lim GZ, Tan KB, Lim JH (2020). An instructive case of amlodipine-induced reversible granulomatous CD30(+) T-cell pseudolymphoma. Australas J Dermatol.

[9] Miguel D, Peckruhn M, Elsner P (2018). Treatment of cutaneous pseudolymphoma: a systematic review. Acta Derm Venereol.

[10] Ploysangam T, Breneman DL, Mutasim DF (1998). Cutaneous pseudolymphomas. J Am Acad Dermatol.

[11] Singh N, Fagan KK, Patel RT, Grider DJ (2023). Pseudolymphoma to lymphoma: a case of chronic reactive lymphoid hyperplasia transforming to primary cutaneous marginal zone lymphoma. Am J Dermatopathol.

